# An Ensemble Semantic Textual Similarity Measure Based on Multiple Evidences for Biomedical Documents

**DOI:** 10.1155/2022/8238432

**Published:** 2022-08-27

**Authors:** Meijing Li, Xianhe Zhou, Keun Ho Ryu, Nipon Theera-Umpon

**Affiliations:** ^1^College of Information Engineering, Shanghai Maritime University, Shanghai 201306, China; ^2^Faculty of Information Technology, Ton Duc Thang University, Ho Chi Minh 700000, Vietnam; ^3^Biomedical Engineering Institute, Chiang Mai University, Chiang Mai, Thailand; ^4^Electrical Engineering Department, Faculty of Engineering, Chiang Mai University, Chiang Mai 50200, Thailand

## Abstract

With the increasing volume of the published biomedical literature, the fast and effective retrieval of the literature on the sequence, structure, and function of biological entities is an essential task for the rapid development of biology and medicine. To capture the semantic information in biomedical literature more effectively when biomedical documents are clustered, we propose a new multi-evidence-based semantic text similarity calculation method. Two semantic similarities and one content similarity are used, in which two semantic similarities include MeSH-based semantic similarity and word embedding-based semantic similarity. To fuse three different similarities more effectively, after, respectively, calculating two semantic and one content similarities between biomedical documents, feedforward neural network is applied to integrate the two semantic similarities. Finally, weighted linear combination method is used to integrate the semantic and content similarities. To evaluate the effectiveness, the proposed method is compared with the existing basic methods, and the proposed method outperforms the existing related methods. Based on the proven results of this study, this method can be used not only in actual biological or medical experiments such as protein sequence or function analysis but also in biological and medical research fields, which will help to provide, use, and understand thematically consistent documents.

## 1. Introduction

With the development of biological and medical fields, the volume of biomedical documents is increasing rapidly. Every year, a big number of papers are published and indexed in PubMed, a standard biomedical document database. By 2022, PubMed comprises more than 34 million biomedical documents. Experts in biology and related fields have made a lot of effort to find necessary documents, and many search technologies are emerging in response to this. In particular, semantically clustering or classifying biomedical documents [1, 2] has always been a very active field. Clustering of medical documents is of great importance to biologists, specialists, and document searchers in all fields of biological research; furthermore, it also greatly facilitates knowledge discovery in a higher level.

In the field of text clustering or retrieval, text similarity measure is a critical step. Text content-based similarity measure is very classical, which was aimed at extracting the keywords as features from the texts [3]. For example, term frequency (TF) or term frequency-inverse document frequency (TF-IDF) is usually applied to extract features and measure the document similarity [4]. In PubMed, the ranking metrics of PubMed-related articles (PMRA) [5] are used to find “related articles” and obtain a collection of articles similar to the search article. PMRA and BM25 [6] have the same theoretical basis to calculate the similarity between biomedical texts based on their contents (headings, abstracts, etc.) by generating item frequencies through Poisson distribution. Obviously, similarity based on text content has the flaw of not capturing the semantic information of the text. In most cases, two texts with the same textual content express different semantic information in different contexts. At this point, semantic text similarity is particularly important.

Semantic similarity of text was firstly applied to vector space model in information retrieval [7]. This model uses semantic similarity between queries and documents to retrieve the documents most relevant to a given query from a collection, for example, web search, subtopic mining, word sense disambiguation, relevance feedback, and text classification [8–10]. Meanwhile, natural language processing (NLP) applications make extensive use of semantic text similarity, including text summarization, machine translation, paraphrasing detection, and sentiment analysis [11]. Semantic similarity among biomedical documents is also very important in information mining in the biomedical field. In the field of medicine, many biomedical words have different meanings in different language context. Therefore, the studies about semantic similarity measure of biomedical document can find the subtle differences between biomedical documents at the semantic level, so as to cluster biomedical documents more accurately.

With the rapid development of neural network for word representation learning [12–14], word embedding has received more and more attention in recent years. Word embedding technology can be applied well in the study of semantic similarity in both general and special fields. Word embedding is a general term for language modeling and representation learning techniques in NLP. Conceptually, it refers to embedding a high dimensional space whose dimension is the number of all words into a continuous vector space of much lower dimension, where each word or phrase is mapped to a vector in the real number field. Methods of word embedding include artificial neural network [15], dimensionality reduction of word cooccurrence matrix [16–18], probability model [19], and explicit representation of the context in which the word resides, etc. Currently, the popular word embedding models mainly include the model of learning context-free words, such as Word2Vec [15] and GloVe [14], and the model of learning context-related words, such as ELMo [20] and BERT [21]. In [22], Word2Vec is applied to calculate the similarity of biomedical terms. In [23], Wu et al. cluster short documents based on semantic similarity applied biterm topic model (BTM) and GloVe. Y. Li et al. recognize Chinese clinical named entities in electronic medical records based on ELMo and lattice long short-term memory model [24]. In [25], semantic similarities between biomedical documents are calculated using BERT algorithm. Although word embedding-based document similarly calculation methods consider the context of the text, they do not consider the professorial knowledge in the biomedical field. Also, these methods still miss biomedical professional relationships between documents.

To solve this weakness, biomedical ontologies are applied to measure the document similarity, such as MeSH and Gene Ontology. MeSH is a standard biomedical ontology published by the National Library of Medicine (NLM), and each article in the MEDLINE database is indexed by several MeSH headings that represent the biomedical domain of the article and summarize the semantic content of the article. Meanwhile, all MeSH headings are organized into a tree structure (MeSH tree) based on semantics. When computing the similarity between articles, the semantics of the articles can be captured by extracting the MeSH features from the article. Therefore, ontology structure-based semantic similarity measure is noticed. There are two kinds of method to measure the similarity between MeSH: one is path-based method, and the other is information content-based method. The similarity based on the paths of the nodes is based on the propagation activation theory [26], which assumes that the hierarchy of the MeSH is organized according to its semantic similarity. Since all headings in the ontology are organized hierarchically, the broader MeSH headings tend to be near the root of the hierarchy and the more specific MeSH headings near the bottom of the hierarchy in the whole MeSH tree. The similarity of nodes in an ontology-based hierarchy depends on the path length (distance) and the depth between nodes. Then, the similarity between nodes of a MeSH heading can be calculated based on their position in the MeSH tree and the depth and distance between them, as in SP [27], WL [28], WP [29], LC [30], Li [31], etc. For the information content of MeSH, it is related to the frequency of MeSH headings in a particular corpus. Meanwhile, MeSH is a tree-like structure, so there may be a relationship between MeSH headings to contain and be contained. Therefore, when counting the number of occurrences of each MeSH heading, it is important to include the number of MeSH headings that have IS-A relationship with a particular MeSH heading. Information content-based similarity calculation methods are applied to measure the relationships between ontology terms such as MeSH heading, which include Lord et al. [32], Resnik [33], Lin [34], and Jiang and Conrath [35]. In [36, 37], they proposed and implement semantic similarity calculation methods based on MeSH ontology for biomedical documents. Ontology-based semantic relationship is applied to other different kinds of fields, such as similarity among functional terms and gene products in chicken [38] and calculation semantic similarity within the knowledge resources in the biomedical field [39], such as Systematized Nomenclature of Medicine-Clinical Terms (SNOMED CT) and Unified Medical Language System (UMLS). However, in the study of similarity of texts in biomedical field, it is not enough to consider only the semantic features embedded in MeSH of medical texts, which is a high generalization of the semantic features of biomedical texts, so it is also essential to consider the semantic features embedded in the textual content of medical texts.

To fully consider the biomedical semantic information in the documents, in this paper, we propose a multi-evidence-based ensemble method. We use vectors from multiple pretrained word embedding models trained in two corpora to represent the semantics of words to capture the word-level semantics in the abstract. For the biomedical semantic information contained in MeSH, we use the MeSH tree to capture the semantic relationships of the MeSH. We also use the traditional TF-IDF to obtain the content features of the text. Finally, we compute the semantic similarity between biomedical texts by fusing multiple features.

The main contributions of this work are as follows:

- Three different kinds of features are extracted and fused by the proposed multi-evidence-based document similarity measurement method, which can be a substantial benefit for understanding semantic information in biomedical documents. We perform a full comparison of the similarity calculation processes and analyze the characteristics of the methods on each feature
- A new ensemble text similarity calculation method based on FNN is proposed to integrate two semantic similarities. A weighted linear combination method is applied to integrate the semantic and content similarities for biomedical documents

## 2. Materials and Methods

### 2.1. Framework

Our proposed method mainly includes three steps: (1) preprocessing, (2) similarity calculation, and (3) similarity integration, as shown in Figure 1. The input is biomedical document data set, and the output is the fusion semantic similarity matrix of the documents. Firstly, three kinds of features are extracted from the documents in preprocessing. Based on extracted features, we measure two semantic similarities and one content similarity between biomedical documents, respectively. Semantic similarities include word embedding-based similarity and MeSH-based similarity. We apply two suitable integrate methods to fuse similarities. We use FNN to generate the semantic similarity matrix. Then, weighted linear combination method is applied to integrate content similarity and semantic similarities.

### 2.2. Preprocessing

To extract multiple features of biomedical texts, we use several different preprocessing methods. In terms of semantic features, we consider the semantic information embedded in the abstract and MeSH. Therefore, given a biomedical document, we first extract the abstract and MeSH terms for the semantic features. For content features, we tokenize the abstract and filter the stopwords. Then, we use TF-IDF method to generate TF-IDF-based content features.

### 2.3. Similarity Calculation

To capture various semantic information, we apply two different kinds of semantic similarity calculation methods, word embedding-based similarity measure and MeSH-based similarity measure. Word embedding-based similarity reflects the context information, and MeSH-based similarity includes semantic information in the biomedical field. TF-IDF-based content similarity is used to reflect the word-level context information in documents.

#### 2.3.1. Word Embedding-Based Semantic Similarity

To obtain the semantic meaning, we use a word embedding model to measure a similarity between texts. Based on the text semantic similarities in the documents, we obtain the semantic similarities between the whole documents.

*(1) Model Training*. Since the research field is the text in the biomedical field, we need a word embedding model trained by corpuses in the biomedical field. To construct a robust model, we used two kinds of large corpora, Wikipedia corpus and MEDLINE corpus. Thus, we can obtain general context information and biomedical professional information together. In this study, Word2Vec [15] is adopted to construct word embedding model, and according to the corpus, the models are named Wiki_W2V and MEDLINE_W2V, respectively. Wiki_W2V represents the model in the general field, and MEDLINE_W2V represents the model in the medical field, and the dimension of word vector in both models is 300 as shown in Table 1.

*(2) Average Semantic Vector of Document*. In general, the more similar the semantic information of two words in the word embedding space are, the greater the dot product between their word vectors. Word2Vec model uses the words as the basic unit to extract semantic information. In this study, we need to extract the semantic information of the whole document. Therefore, we use a method of weighting word vectors in the Word2Vec model to get a semantic vector ASV that can represent document.  Algorithm 1 describes the ASV algorithm in the document.

In Algorithm 1, each document is preprocessed to get *D*_terms_[], and ASV is initialized as an *N*-dimensional zero vector. For each word in *D*_terms_[], if the word exists in vacab of Word2Vec model W2V, the word vector is extracted from the W2V model and added to ASV, and tc_*D*_ is added by 1. After traversing the words of *D*_terms_[], ASV is divided by tc_*D*_.After this step, the vector ASV may be offset in different directions. Therefore, we need to normalize ASV. Here, we choose *Z*-score normalization. Let ASV = [x_1_, x_2_, ⋯, x_n_], Z-score normalization is ASV′ = [*x*_1_′, *x*_2_′, ⋯, *x*_*n*_′], and its changed formula is as follows:

(1) $$\begin{array}{c} x_{i}^{\prime }=\frac{x_{i}-\overset{¯}{x}}{\sigma }, \end{array}$$

where $\overset{¯}{x}$ is the mean and *σ* is the standard deviation.

*(3) Similarity of Document Based on Word Embedding*. Assume that ASV and ASV′ are the average semantic vectors calculated by using Algorithm 1 in document *D* and *D*′, and then, the similarity between documents based on word embedding is expressed as follows:

(2) $$\begin{array}{c} \text{Si}{\text{m}}_{\text{WE}}\left(\text{ASV},\text{AS}{\text{V}}^{\prime }\right)=\frac{\text{ASV}∙\text{AS}{\text{V}}^{\prime }}{\left|\left|\text{ASV}\right|\right|∙\left|\left|\text{AS}{\text{V}}^{\prime }\right|\right|}=\frac{\sum_{i=1}^{n}x_{i}∙{\text{x}}_{i}^{\prime }}{\sqrt{\sum_{i=1}^{n}x_{i}^{2}}\sqrt{\sum_{i=1}^{n}x\prime_{i}^{2}}}, \end{array}$$

where *x*_*i*_ and *x*_*i*_′ are the *i*th elements of the vectors ASV and ASV′, respectively.

#### 2.3.2. MeSH-Based Semantic Similarity

Documents in the MEDLINE database are labeled by a set of MeSH headings (usually 10-15 individuals), which are unified by biomedical experts and represent the subject of the document as shown in Table 2. Therefore, these MeSH headings can represent the semantic information of the document. At the same time, each MeSH heading contains multiple nodes, appearing at different locations in the tree. Each node is represented by a unique tree number see Table 3. Given a set of documents *S* = {*D*_1_, *D*_2_, ⋯, *D*_*n*_}, for each of the reference *D*, the set of MeSH heading marked by it is {*M*_1_, *M*_2_, ⋯, *M*_*n*_}, and then, when calculating the similarity based on MeSH features, we divide it into two steps: (1) calculate the similarity between MeSH heading Sim (*M*, *M*′) and (2) calculate the similarity between documents Sim (*D*, *D*′).

*(1) Similarity of MeSH Heading*. MeSH tree contains 16 subtrees, each of which represents a biomedical direction in terms of medicine. Two path-based methods and two information content-based methods are used to calculate the similarity between nodes, including WP [29], LC [30], Lin [34], and JC [35]. In particular, if two nodes are in two different subtrees, then we can assume that the similarity between the two nodes is 0. Each MeSH heading contains multiple nodes. Therefore, it is necessary to consider that two MeSH headings contain the influence of the degree of similarity between all the nodes. In addition, one MeSH heading may correspond to various nodes in the subtree, and the nodes may be in different subtrees. When we calculate the similarity between two MeSH headings, we usually need to calculate the pairwise similarity between all corresponding nodes and the other node and then take the average value as the final similarity values between two MeSH headings. So, the traditional method may lead to the similarity smaller than the real value. To avoid this problem, we chose average maximum match (AMM). Given two MeSH headings, *M* and *M*′, the similarity between *M* and *M*′ is expressed as follows:

(3) $$\begin{array}{c} \text{Sim}\left(M,M^{\prime }\right)=\frac{\sum_{\text{v}\in \text{M}}\max_{{\text{v}}^{\prime }\in {\text{M}}^{\prime }}\text{Sim}\left(v,v^{\prime }\right)+\sum_{{\text{v}}^{\prime }\in {\text{M}}^{\prime }}\max_{\text{v}\in \text{M}}\text{Sim}\left(v,v^{\prime }\right)}{\left|\text{M}\right|+\left|{\text{M}}^{\prime }\right|}, \end{array}$$

where  max_v′∈M′_Sim(*v*, *v*′) represents the maximum similarity between *v* and any node *v*′ in *M*′.

*(2) Similarity of MEDLINE Document Based on MeSH*. Considering that each document contains multiple MeSH headings and each MeSH heading contains multiple nodes, the similarity from node similarity to MeSH heading is similar to that from MeSH heading similarity to document. Here, we also use AMM method to calculate the similarity of document; given two documents, *D* and *D*′, the similarity between *D* and *D*′ is expressed as

(4) $$\begin{array}{c} \text{Si}{\text{m}}_{\text{MeSH}}\left(\text{D},D^{\prime }\right)=\frac{\sum_{\text{M}\in \text{D}}\max_{{\text{M}}^{\prime }\in {\text{D}}^{\prime }}\text{Sim}\left(M,M^{\prime }\right)+\sum_{{\text{M}}^{\prime }\in {\text{D}}^{\prime }}\max_{\text{M}\in \text{D}}\text{Sim}\left(M,M^{\prime }\right)}{\left|\text{D}\right|+\left|{\text{D}}^{\prime }\right|}. \end{array}$$

Similar to Equation (3), max_M′∈D′_Sim(*M*, *M*′) denotes the maximum similarity between the MeSH heading *M* and any MeSH headings contained in the document *D*′.

#### 2.3.3. Content Similarity

Content similarity refers to the content of MEDLINE document as the characteristic similarity. In this part, a document *D* is represented by a real value vector *C*, which contains the content feature information of *D*. Here, we apply the traditional TF-IDF method to extract the content features of the document. Given documents *D* and *D*′, their corresponding real value vectors are *C* and *C*′, and then, the similarity of documents *D* and *D*′ based on content features can be expressed as

(5) $$\begin{array}{c} {\text{Sim}}_{\text{Con}}\left(D,D^{\prime }\right)=\frac{\text{C}∙{\text{C}}^{\prime }}{\left|\left|\text{C}\right|\right|∙\left|\left|{\text{C}}^{\prime }\right|\right|}. \end{array}$$

### 2.4. Similarity Integration

In the previous part, we generate the document similarity matrix based on one feature, such as word embedding- or MeSH-based semantic features and TF-IDF-based content feature. Based on two integration methods, we integrate the three different document similarities.

#### 2.4.1. Semantic Similarity Integration

To realize the influence of multiple semantic features on the semantic similarity of the document, we apply the feedforward neural network model to integrate the MeSH feature and word embedding feature of the document.

The feedforward neural network model FNN_sem which we constructed for semantic feature integration is shown in Figure 2. The input layer contains 2 input neurons, the hidden layer contains 300 hidden layer neurons, and the output layer contains 1 output neuron. The activation function of the input layer and the hidden layer is ReLU, and the activation function of the output layer is sigmoid.

The purpose of constructing the FNN_sem model is to integrate MeSH features and word embedding features. We take the similarity based on MeSH features, Sim_MeSH_, and similarity based on word embedding, Sim_WE_, as the input and take the semantic similarity based on integration, Sim_Sem_ (similarity after semantic feature integration), as the output. During training, for any two documents *D* and *D*′ in the given data set, if *D* and *D*′ are DR for the same topic, then the similarity between them is set to 0.9; if *D* and *D*′ are PR for the same topic, then it is set to 0.5; otherwise, it is set to 0.1. The number of iterations is set to 100.

After the training, we can input Sim_MeSH_ and Sim_WE_ between documents to get Sim_Sem_, so as to achieve the integration of semantic features.

#### 2.4.2. Fusion Similarity Generation

Weighted linear combination method is applied to integrate the content similarity and semantic similarity. Firstly, Sim_Sem_ and Sim_Con_ normalized processing, making them the minimum value is 0 and the maximum value is 1. Our normalization method choice is SumNorm, whose excellent performance in the treatment of GO term clustering is proved in Zhou et al. [36]. After this, Sim_Sem_ and Sim_Con_ are integrated by linear method. Specifically, setting the weight of Sim_Con_ as *w*, then the similarity after integration is

(6) $$\begin{array}{c} \text{Si}{\text{m}}_{\text{F}}=w∙\text{Si}{\text{m}}_{\text{Con}}+\left(1-w\right)∙\text{Si}{\text{m}}_{\text{Sem}}. \end{array}$$

From Equation (6), we can see that *w* determines the contribution of Sim_Con_ in Sim_F_. When *w* is 0, Sim_F_ is equal to Sim_Sem_. We will find the most appropriate *w* by adjusting the size of *w* to make Sim_Final_ more accurate.

## 3. Experimental Data and Evaluation Methods

In the experiment, we evaluate the performance of the method proposed in this paper. Since there is no official truth value between MEDLINE documents so far, we will evaluate the performance of this method by clustering based on the similarity of this method.

### 3.1. Data

Text REtrieval Conference (TREC) 2005 Genomics Track Data has 4,591,008 MEDLINE database documents (MEDLINE records from 1994 to 2003) and 50 biomedical research topics. The 50 topics simulate real information needs in the biomedical field and are distributed as query headings to all competing information retrieval systems. For each topic, there is absolutely relevant (DR) documents, possibly relevant (PR) documents, and not relevant (NR) documents, where absolutely relevant documents are returned by different retrieval systems, and these documents are then aggregated for manual evaluation by biologists.

In the data obtained above, we need to make further processing, the specific steps are as follows: firstly, we delete the topics with only nine or fewer documents to avoid the occurrence of small clusters because too small clusters affect the fair evaluation results. Then, we further delete the documents related to multiple topics, and finally, we live to 24 topics containing 2,317 documents. In order to fully test the performance of this similarity, we constructed 100 different data sets, each of which randomly selected 3-12 topics and the documents contained in them from 24 topics.  Table 4 shows the basic information of the 100 data sets.

### 3.2. Evaluation Method

The clustering method evaluated in this paper selects spectral clustering algorithm. Many studies have shown [40] that spectral clustering algorithm is an effective and stable clustering method.

#### 3.2.1. Spectral Clustering

Spectral clustering algorithm is very suitable for clustering data with similarity matrix, and it is better than other clustering algorithms in biomedical text clustering. So we use spectral clustering algorithm to perform clustering experiments to investigate the performance of this similarity. The idea of spectral clustering comes from spectral partitioning, which regards data clustering as a multiplexed partitioning problem of undirected graph. The data point is regarded as the vertex *V* of an undirected graph *G* (*V*, *W*), and the set of edge weights *W* = {*S*_*ij*_} represents the similarity between two points calculated based on a certain similarity measure. *S* represents the similarity matrix between data points to be clustered, which is regarded as the adjacency matrix of the undirected graph and contains all the information required for clustering. Then, a partition criterion is defined and optimized so that points within the same class have a high degree of similarity, while points between different classes have a low degree of similarity.

#### 3.2.2. Metrics

In the data obtained by us, the cluster to which each document belongs has been determined, so we can conduct external evaluation by spectral clustering results based on this similarity and the cluster to which they belong. Here, we select four evaluation metrics, which were purity, adjusted Rand index (ARI), normalized mutual information (NMI), and Fowlkes-Mallows index (FMI).

Purity is a simple and transparent assessment standard calculated based on an equation. Each cluster is assigned to the category with the most documents, and accuracy is then measured by correctly counting the number of documents assigned, which is then divided by the total number of documents.

(7) $$\begin{array}{c} \text{Purity}\left(\Lambda ,\text{C}\right)=\frac{1}{N}\overset{k}{\underset{i=1}{\sum }}\underset{j}{\max}\left|\lambda_{i}\cap c_{j}\right|, \end{array}$$

where *Λ* = {*λ*_1_, *λ*_2_, ⋯, *λ*_*i*_, ⋯, *λ*_*n*_} represents the true value set of the cluster, *C* = {*c*_1_, *c*_2_, ⋯, *c*_j_, ⋯, *c*_*n*_} represents the clustering of clustering results, and *N* represents the total number of references.

Rand index (RI) calculates the similarity measure between the two clusters by considering all sample pairs and calculating the pairs allocated in the same or different clusters in the predicted and real clusters, and its value range is 0 to 1.

(8) $$\begin{array}{c} \text{RI}=\frac{\text{TP}+\text{TN}}{\text{TP}+\text{FP}+\text{TN}+\text{FN}}, \end{array}$$

where TP is the number of documents in both a class and a cluster, FP is the number of documents in a class but not in a cluster, TN is the number of documents in different classes but in a cluster, and FN is the number of documents in different classes and in different clusters.

Adjusted Rand index (ARI) is an improvement on RI and was proposed by Hubert and Arabie in 1985 [41]. Since the problem with RI is the division of two random variables, its RI value is not a constant close to 0. Adjust the Rand coefficient to assume that the super distribution of the model is a random model; that is, the division of *X* and *Y* is random, and then, the number of data points of each category and cluster is fixed, and its value range becomes -1 to 1. The larger the model, the better the effect:

(9) $$\begin{array}{c} \text{ARI}=\frac{\text{RI}-\text{E}\left(\text{RI}\right)}{\max\left(\text{RI}\right)-\text{E}\left(\text{RI}\right)}, \end{array}$$

where E(RI) is the expected value of RI.

NMI is used to measure the degree of correspondence between the two data distributions. In the study of Ghosh [42], it was found that NMI index could achieve a good evaluation effect of clustering. Therefore, we also use NMI to evaluate the performance of clustering:

(10) $$\begin{array}{c} \text{NMI}=\frac{I\left(P;Q\right)}{\sqrt{H\left(P\right)∙H\left(Q\right)}}, \end{array}$$

(11) $$\begin{array}{c} =\frac{\sum_{i,j}n_{i,j}\log\left(n∙n_{i,j}/n_{i}n_{j}\right)}{\sqrt{\left(\sum_{i}n_{i}\log\left(n_{i}/n\right)\right)\left(\sum_{j}n_{j}\log\left(n_{j}/n\right)\right)}}. \end{array}$$

In Equation (10), *P* and *Q* are predicted labels after clustering and correct labels, respectively, *I*(*P*; *Q*) represents their mutual information, *H*(*P*) is the entropy of *P*, and *H*(*Q*) is the entropy of *Q* [40], which can be written into Equation (11) according to Equation (10). In Equation (11), *n* is the total number of documents in the data set, *n*_*i*_ is the number of documents in the correct class *i*, *n*_*j*_ is the number of documents in the predicted cluster *j*, and *n*_*i*,*j*_ is the total number of documents in both class *i* and cluster *j*.

FMI was proposed by Fowlkes and Mallows [43] in 1983 as the geometric mean of the pairwise precision and recall for document pairs:

(12) $$\begin{array}{c} \text{FMI}=\frac{\text{TP}}{\sqrt{\left(\text{TP}+\text{FP}\right)∙\left(\text{TP}+\text{FN}\right)}}, \end{array}$$

where TP, FP, and FN have the same meaning as expressed in RI.

## 4. Experiment Result and Discussion

To fully evaluate the performance of each similarity mentioned in this paper, we set up three groups of clustering experiments.

### 4.1. The Analysis of the Result Based on Single Similarity

To find the best calculation method based on each single feature, we set up a clustering experiment based on a single similarity, including (1) methods based on word embedding features, WE_M (model MEDLINE_W2V as word embedding model) and WE_W (model WIKI_W2V as word embedding model); (2) methods based on MeSH features include LC [30], WP [29], Lin [34], and JC [35] (In the JC method, the value of *λ* is changed to determine the optimal result of the method); and (3) content-based method, Con.

The clustering results of 100 data sets based on the computing method of similarity of word embedding feature and MeSH feature are shown in Tables 5 and 6, respectively, with the maximum shown in italics. As can be seen from Table 5 and Figure 3(a), in the similarity based on word embedding features, the clustering effect of WE_M method (purity = 0.810, ARI = 0.499, NMI = 0.600, and FMI = 0.634) is better than that of WE_W (purity = 0.705, ARI = 0.306, NMI = 0.412, and FMI = 0.493), indicating that the overall effect of MEDLINE_W2V model was better than that of Wiki_W2V model. As can be seen from Table 6 and Figure 4, among the clustering methods based on MeSH features, the overall effect of JC method was the best, especially when *λ* = 1 (purity = 0.834, ARI = 0.668, NMI = 0.670, and FMI = 0.762), and the overall effect of LC method (purity = 0.788, ARI = 0.453, NMI = 0.536, and FMI = 0.599) was the worst. In addition, it can be seen from Figure 4 that all methods have little difference in each evaluation methods, and the average value of JC method in all evaluation methods is the highest. This shows that all the methods have little difference in the effects of data sets with different sizes and proves the superiority of JC method in MeSH feature-based methods again.

We also compared the methods that achieved the best clustering results based on the similarity of each feature, and the comparison results are shown in Table 7 and Figure 3(b), with the maximum shown in italics. Overall, when *λ* = 1, the JC method achieves the maximum values of purity and FMI, which are 0.834 and 0.762, respectively. The maximum values of ARI and NMI obtained by Con were 0.701 and 0.738, respectively. The experimental results show that the semantic similarity based on MeSH feature is better than that based on word embedding feature. Meanwhile, the effect of semantic similarity based on MeSH feature is similar to that of content similarity based on content feature. On the other hand, it was confirmed that the effect of the semantic similarity according to the MeSH feature was similar to that of the content similarity according to the content feature.

### 4.2. The Analysis of the Result Based on Semantic Similarity

We conduct a clustering experiment by integrating the similarity of MeSH and word embedding features to explore the optimal combination mode. There are four methods based on the MeSH feature, and the value of *λ* in the JC method is set from 1 to 5. There are a total of 8 similarity degrees, and two methods based on the word embedding feature are WE_M and WE_W, respectively, so 16 combinations of pair-combined methods are generated, based on Table 8.

The clustering results of similarity on 100 data sets based on the combination of MeSH and word embedding features are shown in Table 8, with the maximum shown in italics. From Table 8, we can see that the overall clustering effect of semantic similarity after integration is generally higher than that of a single similarity. For example, the average values of all metrics (purity = 0.859, ARI = 0.622, NMI = 0.702, and FMI = 0.727) after the combination of LC method and WE_M method are all higher than that of LC (purity = 0.788, ARI = 0.453, NMI = 0.536, and FMI = 0.599). At the same time, we find that the clustering effect of all the methods based on MeSH combined with WE_M method is higher than that of the method combined with WE_W method, which fully shows that the clustering effect of WE_M method is better than that of WE_W method. Overall JC method had the best efficacy in *λ* = 1 and the combination effect of WE_M method (purity = 0.896, ARI = 0.738, NMI = 0.779, and FMI = 0.813), while WP method and WE_W method (purity = 0.808, ARI = 0.529, NMI = 0.606, and FMI = 0.665) had the worst. Therefore, my next experiment will use the combination of JC (*λ* = 1) method and WE_M method (JC_1_WE_M method) to calculate semantic similarity.

### 4.3. The Analysis of the Result Based on Fusion Similarity

As mentioned in the method, semantic similarity and content similarity are integrated by weighted linear combination method. For example, JC_1_WE_M method is used to calculate semantic similarity as mentioned above, and Con method is used to calculate similarity based on content features. According to Equation (6), we adjust the value of *w* to find the best value of *w*.

In combination with Table 9 and Figure 5, we can see that with the increasing value of *w*, the average of all metrics slowly increased and the standard deviation slowly decreased and reached a peak value when *w* = 0.7. The average (purity = 0.947, ARI = 0.818, NMI = 0.878, and FMI = 0.866) reached the maximum, and the standard deviation (purity = 0.049, ARI = 0.169, NMI = 0.098, and FMI = 0.125) reached the minimum. It shows that the similarity based on content features has a great influence on the results. Compared with semantic similarity, through the integration of semantic similarity and content similarity, the average value of each metric is significantly improved and the standard deviation is significantly reduced, indicating that the more features considered, the better the clustering effect.

### 4.4. Comparison with Related Work

In order to fully verify the clustering performance of our proposed similarity, we compare it with the previous correlation clustering methods.  Table 10 shows the index comparison results of the similarity proposed by us (Sim_0.7_, that is, the similarity at *w* = 0.7) and clustering method proposed by Zhu et al. [37] on the same data set.

The clustering method proposed by Zhu et al. is based on the linear integration of MeSH feature similarity and content feature similarity to carry out spectral clustering experiments. From Table 10, it can be clearly seen that the average values of all metrics of similarity proposed in this paper in spectral clustering are higher than method of Zhu et al. In particular, the improvement was particularly significant in the FMI (increased 0.061). This result further demonstrates the validity of our proposed similarity by integrating multiple MEDLINE documents features.

### 4.5. Discussion for Interpretability of Proposed Method

The research of text similarity can generally extract features from two aspects: one is the content of the text, and the other is the semantics of the text. At the same time, texts in special fields often contain semantic features unique to the field, and we also need to extract such features. In addition, for one aspect of feature extraction, the number considered often determines the performance of similarity. In the previous studies, there are two kinds of defects: one [5, 6] is that only the content is considered without considering the semantic aspect, and the other [37] is that the number of features considered in one aspect is less.

Our method makes up for the above two defects at the same time, which is we consider the content and semantic features of the biomedical documents at the same time. On this basis, we consider multiple features in the semantic aspect (extracted from MeSH and extracted from the text content through word embedding) and fuse them, so as to improve the performance of biomedical text similarity. In the experimental part, we first screened out the best calculation methods in terms of semantics and content, as shown in Tables 5, 6, and 7. Then, we fuse the two semantic features through FNN to screen the optimal semantic fusion scheme, as shown in Table 8. Finally, the content and semantic aspects are fused through the linear model, as shown in Table 10 to obtain the final similarity calculation method.

Furthermore, our experimental results prove that our proposed multi-evidence-based semantic text similarity calculation method enhances the biomedical document clustering effort when compared to various existing methods; it has shown superior performances in several evaluation metrics such as purity, ARI, NMI, and FMI. Essentially, our proposed method extracts and fused different features that findings are able to represent semantic information of the biomedical documents.

## 5. Conclusion

With multiple documents, the similarity calculation has limitations in terms of accuracy. Therefore, to solve the problems, in this paper, we proposed a new semantic similarity of MEDLINE documents by extracting the semantic information contained in the MeSH title and abstract from the MEDLINE document and combining the content information. In this proposed method, after calculating semantic similarity and content similarity between medical documents, FNN and weighted linear combination method were applied to integrate semantic and content similarity. In addition, the proposed method was compared with the existing basic methods for analyzing medical documents. The experimental results showed that the clustering effect was significantly improved as the number of features considered as semantic similarity integration increased with the semantic similarity integration of the integrated MeSH function and the word embedding function from a single similarity, and the content similarity and clustering performance were correlated in each clustering metric. It was confirmed that the multievidence method outperforms the traditional methods.

One of the strong points of this study is that it achieves the purpose of performance improvement by considering and integrating various semantic features. Our proposed method is based on the idea of multifunctional convergence, which can play an important role not only in experts in biomedical experts and information mining in general fields. Therefore, the research method of clustering these multiple features can be applied to other fields of similarity research, such as a study to calculate the similarity between genes. At the same time, in the general domain, if the study subject contains multiple features, we can apply this idea to improve performance.

## Figures and Tables

**Figure 1:** Workflow of proposed method.

**Figure 2:** Illustration of FNN_sem.

**Figure 3:** Mean and standard deviation of evaluation metrics. (a) Clustering results based on two word embedding based similarities; (b) Clustering results based on three different similarities.

**Figure 4:** Statistical significance test of cluster results. (a) Purity scores; (b) ARI scores;(c) NMI scores; (d) FMI scores.

**Figure 5:** Metrics for spectral clustering based on final similarity in different w. (a) Average value of cluster metrics; (b) Standard deviation of cluster metrics.

**Algorithm 1:** Algorithm of *ASV* calculation.

**Table 1:** The details of two embedded models.

Model	Dimension	Vocabulary size	Corpus
Wiki_W2V	300	3,000,000	Wikipedia
MEDLINE_W2V	300	2,000,000	MEDLINE

**Table 2:** A MEDLINE document and its related MeSH terms.

PMID	MeSH term
12625756	Animals
	DNA
	Drug delivery system
	Electroporation
	Gene transfer techniques
	Humans
	Neoplasms

**Table 3:** Two MeSH terms and their tree numbers.

MeSH term	MeSH tree number
Melanosomes	A11.284.430.214.190.500.560
	A11.284.430.214.190.875.190.190.560
	A11.409.750.560
	A11.436.265.531.560
	A11.436.613.560
Sarcomeres	A10.690.552.875.700
	A11.284.430.214.190.875.820
	A11.620.249.850.700
	A11.620.500.500.700

**Table 4:** Description of the data set.

	cluster_num	doc_num_cluster	doc_num_data
Min	3	10	84
Max	12	385	1541
Average	6.9	88.4	609.4

Note: cluster_num represents the number of clusters in the 100 data sets, doc_num_cluster represents the number of documents contained in each cluster, and doc_num_data represents the number of documents contained in each data set.

**Table 5:** Metrics (average ± SD) of all 100 data sets for spectral clustering based on word embedding.

Method	Purity	ARI	NMI	FMI
**WE_M**	**0.810 ± 0.081**	**0.499 ± 0.185**	**0.600 ± 0.128**	**0.634 ± 0.149**
WE_W	0.705 ± 0.093	0.306 ± 0.112	0.412 ± 0.114	0.493 ± 0.144

**Table 6:** Metrics (average ± SD) of all 100 data sets for spectral clustering based on MeSH semantic similarity, where JC_i: JC with *λ* = i.

Method	Purity	ARI	NMI	FMI
LC	0.788 ± 0.085	0.453 ± 0.156	0.536 ± 0.112	0.599 ± 0.139
WP	0.794 ± 0.088	0.472 ± 0.167	0.554 ± 0.117	0.613 ± 0.145
Lin	0.830 ± 0.083	0.570 ± 0.184	0.629 ± 0.130	0.683 ± 0.149
**JC_1**	**0.834 ± 0.092**	**0.668 ± 0.181**	**0.670 ± 0.135**	**0.762 ± 0.142**
JC_2	0.824 ± 0.081	0.561 ± 0.178	0.617 ± 0.128	0.681 ± 0.141
JC_3	0.821 ± 0.077	0.545 ± 0.168	0.605 ± 0.118	0.669 ± 0.136
JC_4	0.812 ± 0.080	0.513 ± 0.163	0.584 ± 0.117	0.645 ± 0.135
JC_5	0.801 ± 0.082	0.492 ± 0.153	0.563 ± 0.110	0.629 ± 0.134

**Table 7:** Comparison of metrics (average ± SD) for spectral clustering in all 100 data sets based on the similarity of different features.

Method	Purity	ARI	NMI	FMI
WE_M	0.810 ± 0.081	0.499 ± 0.185	0.600 ± 0.128	0.634 ± 0.149
JC_1	**0.834 ± 0.092**	0.668 ± 0.181	0.670 ± 0.135	**0.762 ± 0.142**
Con	0.813 ± 0.087	**0.701 ± 0.143**	**0.738 ± 0.102**	0.724 ± 0.162

**Table 8:** Metrics (average ± SD) of all 100 data sets for spectral clustering based on 16 integrated semantic similarities.

Method	Purity		ARI		NMI		FMI	
	WE_M	WE_W	WE_M	WE_W	WE_M	WE_W	WE_M	WE_W
LC	0.859 ± 0.079	0.834 ± 0.081	0.622 ± 0.193	0.572 ± 0.189	0.702 ± 0.127	0.642 ± 0.131	0.727 ± 0.145	0.692 ± 0.147
WP	0.844 ± 0.091	0.808 ± 0.092	0.612 ± 0.197	0.529 ± 0.168	0.690 ± 0.129	0.606 ± 0.126	0.723 ± 0.149	0.665 ± 0.149
Lin	0.860 ± 0.096	0.849 ± 0.111	0.668 ± 0.209	0.672 ± 0.217	0.725 ± 0.137	0.708 ± 0.150	0.765 ± 0.153	0.770 ± 0.157
JC_1	**0.896 ± 0.074**	0.868 ± 0.097	**0.738 ± 0.179**	0.706 ± 0.197	**0.779 ± 0.120**	0.734 ± 0.143	**0.813 ± 0.131**	0.794 ± 0.141
JC_2	0.868 ± 0.096	0.846 ± 0.105	0.686 ± 0.209	0.643 ± 0.213	0.736 ± 0.138	0.684 ± 0.147	0.776 ± 0.154	0.745 ± 0.160
JC_3	0.863 ± 0.087	0.853 ± 0.097	0.662 ± 0.199	0.651 ± 0.208	0.720 ± 0.131	0.695 ± 0.144	0.756 ± 0.150	0.749 ± 0.159
JC_4	0.854 ± 0.085	0.843 ± 0.088	0.635 ± 0.196	0.642 ± 0.188	0.700 ± 0.128	0.692 ± 0.117	0.739 ± 0.146	0.724 ± 0.135
JC_5	0.850 ± 0.084	0.818 ± 0.079	0.623 ± 0.196	0.549 ± 0.179	0.691 ± 0.129	0.614 ± 0.122	0.730 ± 0.145	0.676 ± 0.142

**Table 9:** Metrics (average ± SD) of all 100 data sets for spectral clustering based on final similarity in different *w*.

*w*	Purity	ARI	NMI	FMI
0.1	0.904 ± 0.067	0.749 ± 0.177	0.790 ± 0.117	0.820 ± 0.131
0.2	0.903 ± 0.075	0.743 ± 0.188	0.793 ± 0.121	0.815 ± 0.137
0.3	0.913 ± 0.063	0.760 ± 0.179	0.806 ± 0.116	0.826 ± 0.131
0.4	0.915 ± 0.068	0.757 ± 0.184	0.814 ± 0.115	0.822 ± 0.137
0.5	0.920 ± 0.067	0.767 ± 0.183	0.825 ± 0.112	0.830 ± 0.137
0.6	0.927 ± 0.064	0.785 ± 0.176	0.840 ± 0.107	0.843 ± 0.131
**0.7**	**0.947 ± 0.049**	**0.818 ± 0:169**	**0.887 ± 0:098**	**0.866 ± 0:125**
0.8	0.941 ± 0.057	0.809 ± 0.174	0.869 ± 0.100	0.860 ± 0.130
0.9	0.933 ± 0.063	0.791 ± 0.180	0.852 ± 0.106	0.866 ± 0.133

**Table 10:** Comparison of metrics (average ± SD) between the similarities proposed in this paper and the method of Zhu et al. in spectral clustering.

Method	Purity	ARI	NMI	FMI
**Sim**_**0.7**_	**0.947 ± 0.049**	**0.818 ± 0.169**	**0.887 ± 0.098**	**0.866 ± 0.125**
Zhu et al.	0.924 ± 0.048	0.797 ± 0.179	0.866 ± 0.104	0.805 ± 0.136

## Data Availability

The datasets used to support the findings of this study are available from the corresponding author upon request.
